This article has been retracted.

# MicroRNA-153 is a prognostic marker and inhibits cell migration and invasion by targeting SNAI1 in human pancreatic ductal adenocarcinoma

**DOI:** 10.3892/or.2015.4051

**Published:** 2015-06-11

**Authors:** ZHENGHAI BAI, JIANGLI SUN, XIAOBO WANG, HAI WANG, HONGHONG PEI, ZHENGLIANG ZHANG

**Affiliations:** Department of Emergency, The Second Affiliated Hospital of Xi’an Jiaotong University, Xi’an, Shaanxi 710004, P.R. China

**Keywords:** microRNA-153, PDAC, prognosis, SNAI1, tumor metastasis

## Abstract

Human pancreatic ductal adenocarcinoma (PDAC) is an aggressive cancer type with early metastasis, which leads to poor prognosis for patients. Mounting evidence suggests that microRNAs (miRNAs) act as critical factors for tumor recurrence and metastasis. miR-153 has been suggested as a novel tumor-associated miRNA, which is involved in tumor metastasis. However, the clinical significance of miR-153 and its role in PDAC remains to be investigated. The aim of the present study was to investigate the expression levels of miR-153 using RT-qPCR in human PDAC cell lines and tissues. A clinical association analysis was performed to investigate the clinical significance of miR-153. The results showed that, the relative expression of miR-153 in PDAC cells was obviously decreased as compared to that in the normal human pancreatic duct epithelial cell line. The mean expression of miR-153 in PDAC tissues was significantly reduced as compared to that in the normal pancreatic tissues. The clinical analysis revealed that a low expression of miR-153 was closely associated with poor prognostic features and shorter long-term survival of PDAC patients. Furthermore, univariate and multivariate Cox regression analyses showed that miR-153 was an independent prognostic factor for predicting survival in PDAC patients. *In vitro* studies demonstrated that the upregulation of miR-153 inhibited migration and invasion in MIAPaCa-2 cells. By contrast, the downregulation of miR-153 increased the number of migrated and invaded AsPC-1 cells. miR-153 inversely regulated SNAI1 abundance in MIAPaCa-2 cells. Notably, SNAI1 was identified as a direct target of miR-153 in PDAC. Furthermore, an inverse correlation between miR-153 and SNAI1 expression was observed in PDAC tissues. In conclusion, the results showed miR-153 is an independent prognostic marker for predicting survival in PDAC patients and inhibits cell migration and invasion by targeting SNAI1.

## Introduction

Pancreatic ductal adenocarcinoma (PDAC) is an aggressive type of cancer with early metastasis and is usually diagnosed at late stage due to lack of specific symptoms (1). Accumulating evidence has shown that the deregulation of microRNAs (miRNAs) is observed in PDAC, some of which function as tumor-suppressor genes or oncogenes (2).

The expression of miR-153 in glioblastoma (GBM) is significantly lower than that in non-neoplastic brain tissue. miR-153 inhibits cell proliferation and induces apoptosis by targeting B-cell lymphoma 2 (Bcl-2) and myeloid cell leukemia sequence-1 (Mcl-1) in GBM cells (3–9). A reduced expression of miR-153 has been observed in ovarian tumors and its low expression is correlated with FIGO grade 3 and advanced clinical stage, suggesting it is of potential importance as a diagnostic biomarker (10). miR-153 sensitizes leukemia cells to As2O3-induced apoptosis (11). The down-regulation of miR-153 promotes epithelial-mesenchymal transition (EMT) via SNAI1 and ZEB2. Results of a clinical analysis have indicated that a low expression level of miR-153 was significantly associated with metastasis and poor prognosis in oral cancer patients (12). In breast cancer, miR-153 reduces cell proliferation and viability and induces apoptosis in MDA-MB-231 cells (13). miR-153 expression is significantly lower in lung cancer tissues as compared with adjacent tissues and exerted antitumor activity in lung cancer by targeting protein kinase B (AKT) (14). Furthermore, miR-153 reduced the number of migrated and invaded non-small-cell lung cancer (NSCLC) cells by targeting the dynamic change of adamalysin 19 (ADAM19) (15). The above mentioned studies indicate that miR-153 is a tumor suppressive miRNA. However, miR-153 was found to be overexpressed in endome-trial, prostate and colorectal cancer (16–18). Overexpression of miR-153 promoted cell cycle transition and cell proliferation by inhibiting phosphatase and tensin homolog deleted on chromosome 10 (PTEN) in prostate cancer (17). miR-153 promoted invasiveness indirectly by inducing matrix metal-loprotease enzyme 9 (MMP9) production, whereas drug resistance was mediated directly by inhibiting the forkhead transcription factor forkhead box O3a (FOXO3a) (18). Therefore, the functional significance of miR-153 in cancer development and progression seem to be cancer-type specific. However, the clinical and prognostic significance of miR-153 in human PDAC has not been elucidated.

In the present study, the expression levels of miR-153 were measured by RT-qPCR in human PDAC cell lines and tissues. A clinical association analysis was performed to investigate the clinical significance of miR-153. Furthermore, the prognostic value of miR-153 was determined by the Kaplan-Meier estimation. Our results showed that an impaired expression of miR-153 was observed in PDAC and it may be a potential prognostic biomarker for PDAC patients.

## Materials and methods

### Clinical samples and cell lines

The patients included 27 males and 53 females, who underwent resection of their PDAC in the Department of General Surgery at the Second Affiliated Hospital of Xi’an Jiaotong University between January 2005 and December 2010, with a median follow-up time of 18.7 months. The patients did not receive preoperative chemotherapy or radiotherapy. The stage of cancer was determined according to the Cancer Staging System of the Union for International Cancer Control (UICC, 2002). The demographic features and clinicopathological data are shown in Table I. Thirty normal pancreatic tissue samples were also obtained from the patients who underwent pancreatoduodenectomy or distalpancreatectomy for diseases other than pancreatic cancer. The samples were used after informed consent was obtained. The Xi’an Jiaotong University Ethics Committee approved all the protocols according to the Declaration of Helsinki (as revised in Tokyo, 2004).

A normal human pancreatic duct epithelial cell line (HPDE6-C7) and five PDAC cell lines (PANC-1, MIAPaCa-2, BxPC-3, AsPC-1 and PL45) were purchased from the Institute of Biochemistry and Cell Biology, Chinese Academy of Sciences, (Shanghai, China). The cells were cultured in complete Dulbecco’s modified Eagle’s medium (DMEM) containing 10% fetal bovine serum (FBS) (both from Gibco, Grand Island, NY, USA) with 100 U/ml penicillin and 100 *µ*g/ml streptomycin (Sigma, St. Louis, MO, USA) in a humidified container of 5% CO_2_ incubator at 37°C.

### Immunohistochemical staining

Immunohistochemistry was performed on paraformaldehyde-fixed paraffin sections. SNAI1 (ab117866; Abcam, Cambridge, MA, USA) antibody was used in immunohistochemistry with the streptavidin peroxidase-conjugated (SP-IHC) method. Immunohistochemistry was performed as previously described (19). The percentage of positive cells was graded as per the following criteria: 0, <10%; 1, 10–30%; 2, 31–50% and 3, >50%.

### Real-time reverse transcription-quantitative PCR (RT-qPCR)

The expression of miR-153 in 80 cases of PDAC tissues was determined by RT-qPCR. Total RNA was isolated from gastric cancer cells using TRIzol^®^ reagent (Invitrogen-Life Technologies, Carlsbad, CA, USA) according to the manufacturer’s instructions. Total RNA was reverse-transcribed using RevertAid™ First Strand cDNA Synthesis kit (Thermo Fisher Scientific, Inc., Waltham, MA, USA) according to the manufac turer’s instructions. The PCR amplification for the quantification of miR-153 and U6 was performed using a MicroRNA Reverse Transcription kit and TaqMan Human MiRNA Assay kit (both from Applied Biosystems, Foster City, CA, USA). The median value of miR-153 expression was considered as the threshold. MiR-153 high: value of expression > the median value; miR-153 low: value of expression < the median value. The relative expression of miR-153 was shown as the fold difference relative to U6 (20).

Primer pairs against *Homo sapiens* gene SNAI1 (HP208950) and GAPDH (HP205798) were purchased from OriGene (Beijing, China). The PCR amplification for the quantification of the SNAI1 and GAPDH mRNAs was performed using an ABI PRISM 7300 Sequence Detection system (Applied Biosystems) and a SYBR® Premix Ex *Taq*™ II (Perfect Real-Time) kit (Takara Bio, Shiga, Japan), as previously described (21).

### Plasmids and cell transfection

miRNA vectors, including miR-153 expression vector (HmiR0039-MR04), the control vector for miR-153 (CmiR0001-MR04), miR-153 inhibitor (HmiR-AN0214-AM04) and the negative control for the miR-153 inhibitor (CmiR-AN0001-AM04) were purchased from GeneCopoeia (Guangzhou, China). The cells were transfected with the vectors mentioned above using Lipofectamine 2000 according to the manufacturer’s instructions (Invitrogen) (20).

### Western blotting

The primary antibodies used in the immunoblotting assays were: SNAI1 (ab117866; Abcam) and GAPDH (G8140; United States Biological, Swampscott, MA, USA). Horseradish peroxidase-conjugated secondary antibody (Bio-Rad, Hercules, CA, USA) was used at a 1:1,000–1:5,000 dilution and detected using a Western Blotting Luminol Reagent (sc-2048; Santa Cruz Biotechnology, Inc., Santa Cruz, CA, USA), as described in a previous study (22).

### Boyden chamber and Transwell invasion assays

PDAC cells were resuspended with reduced serum DMEM medium and the density was adjusted to 2.5×10^5^/ml. A 200 *µ*l cell suspension was added into the upper chamber and 750 *µ*l DMEM medium containing 10% FBS was added into the lower chamber. A Boyden chamber assay (Neuro Probe, Gaithersburg, MD, USA) was used to analyze PDAC cell migration, as previously described (23). Transwell invasion assays were carried out in 6-well plates with Transwell inserts equipped with 8-*µ*m pores (Nalge Nunc International Corp., Naperville, IL, USA) coated with Matrigel at 1:6 dilution (Becton-Dickinson Labware, Bedford, MA, USA) as previously described (24).

### Luciferase reporter assay

The 3′-untranslated region (3′-UTR) sequence of SNAI1, predicted to interact with miR-153 or a mutated sequence within the predicted target sites, was produced and inserted into the *Xba*I and *Fse*I sites of the pGL3 control vector (Promega, Madison, WI, USA). These constructs were designated as wild-type (wt) SNAI1–3′-UTR or mutant (mt) SNAI1–3′-UTR, respectively. For the reporter assay, MIAPaCa-2 cells were seeded in 24-well plates and transfected with the above constructs and miR-153 expression vector, miR-153 inhibitor, control vector or negative control. After 48 h, the cells were collected and *Renilla* luciferase activity was measured using the Dual-Luciferase Reporter Assay System (Promega) according to the manufacturer’s instructions. Results were obtained from three independent experiments performed in duplicate.

### Statistical analysis

Results are presented as mean ± SEM. Significance was established, with the SPSS statistical package for Windows version 13 (SPSS, Inc., Chicago, IL, USA) and GraphPad Prism 5 software (GraphPad Software, Inc., San Diego, CA, USA), using a Pearson’s Chi-square test, a Kaplan-Meier plot, a log-rank test, the multi-variant Cox regression analysis, Pearson’s correlation coefficient or a two-tailed Student’s t-test when appropriate. Differences were considered significant at P<0.05.

## Results

### Expression of miR-153 in human PDAC cells and tissue samples

Initially, we assessed the expression of miR-153 in a normal human pancreatic duct epithelial cell line (HPDE6-C7) and five PDAC cell lines (PANC-1, MIAPaCa-2, BxPC-3, AsPC-1 and PL45). As measured by RT-qPCR, the relative expression of miR-153 in PDAC cell lines was significantly lower than that in the HPDE6-C7 (P<0.05, Fig. 1A). We then determined the expression of miR-153 in 80 cases of PDAC tissues and 30 cases of normal pancreas tissues. Quantitative analysis indicated that the mean level of miR-153 in PDAC tissues was obviously lower as compared with that in normal pancreas tissues (P<0.05), (Fig. 1B). Thus, the expression of miR-153 was impaired in PDAC.

### Clinical significance of miR-153 in PDAC patients

The expression of miR-153 was considered as either low (n=40) or high (n=40) according to the cut-off value, which was defined as the median of the cohort. The association between miR-153 expression and clinicopathological variables of PDAC patients are presented in Table I. Results of the statistical analysis revealed that, miR-153 was expressed at prominent lower levels in patients with lymph node metastasis, tumor recurrence, poor tumor differentiation and advanced tumor stage (P<0.05, respectively). The Kaplan-Meier survival analysis was performed to determine the prognostic value of miR-153 in PDAC patients. PDAC patients with a low expression of miR-153 had an evidently lower 3-year overall survival (OS) as compared with those with a high expression of miR-153 (P=0.041, Fig. 2). Furthermore, it was shown that patients with a low expression of miR-153 were associated with shorter recurrence-free survival (RFS) (P=0.039, Fig. 2). In addition, a univariate Cox regression analysis indicated that clinicopathological characteristics, including tumor differentiation and stage, lymph node metastasis, tumor recurrence and miR-153 expression, were significantly associated with OS (P<0.05, respectively, Table II). Notably, the multivariate Cox regression analysis indicated that miR-153 expression was an independent factor for predicting the 3-year OS of PDAC patients (P=0.038, Table II). These data indicated that miR-153 is a potent biomarker for predicting the prognosis of PDAC patients.

### miR-153 inhibits PDAC cell migration and invasion in vitro

To investigate the role of miR-153 in PDAC, miR-153 was upregulated in the MIAPaCa-2 PDAC cell line via expression of plasmid transfection. As assessed by RT-qPCR, the expression of miR-153 was overexpressed by miR-153 expression vector in MIAPaCa-2 cells (P<0.05, Fig. 3A). Boyden chamber assays were performed to determine the effect of altering miR-153 levels on tumor cell migration. We found that upregulation of miR-153 led to a significant reduction of cell migration in MIAPaCa-2 cells (P<0.05, Fig. 3B). Furthermore, as determined by Transwell invasion assays, the number of invaded MIAPaCa-2 cells was significantly decreased after miR-153 overexpression (P<0.05, Fig. 3B). miR-153 downregulated AsPC-1 cells, which was confirmed by RT-qPCR (P<0.05, Fig. 3C). As expected, downregulation of miR-153 obviously promoted AsPC-1 cell migration and invasion (P<0.05, respectively, Fig. 3D). Thus, miR-153 inhibited cell migration and invasion in PDAC.

### SNAI1 is identified as a functional target of miR-153 and is downregulated in PDAC specimens

Additional studies were performed to identify the molecular mechanisms by which miR-153 inhibited cell migration and invasion in PDAC. Previous studies reported that miR-153 was a novel regulator of EMT by targeting SNAI1 and ZEB2 in human epithelial cancers (12). MIAPaCa-2 cells that were transfected with miR-153 and control vectors were subjected to RT-qPCR and western blotting for SNAI1 expression. SNAI1 mRNA and protein levels were significantly reduced by upregulation of miR-153 in MIAPaCa-2 cells (P<0.05, respectively, Fig. 4A and B). To further demonstrate that SNAI1 was directly targeted by miR-153 in PDAC cells, we investigated whether the miR-153 directly interacted with the 3′-UTR of SNAI1 mRNA using a dual-luciferase reporter assay. miR-153 signifi-cantly inhibited the luciferase activity of SNAI1 containing a wt 3′-UTR, but did not suppress the activity of SNAI1 with a mt 3′-UTR (P<0.05, Fig. 4C and D). When anti-miR-153 was transfected, an increase in luciferase activity of wt SNAI1 3′-UTR was observed. However, no relative increase in activity was identified following transfection with the mt SNAI1 3′-UTR constructs (P<0.05, Fig. 4C and D). Thus, our data strongly suggested that SNAI1 is a target of miR-153 in PDAC.

Expression of SNAI1 was detected by immunohisto-chemistry in the previous cohort of 80 cases of PDAC tissues and 30 cases of normal pancreas tissues. The mean level of SNAI1 protein was demonstrated to be significantly higher in PDAC tissues as compared with the normal pancreas tissues (P<0.05, Fig. 5A). SNAI1 immunoreactivity was considered as either negative (score 0) or positive (scores 1–3). In these cases, SNAI1 expression was detected in 75.0% (30/40) of the PDAC samples with a low expression of miR-153, whereas only 42.5% (17/40) of the PDAC specimens with a high expression of miR-153 showed a positive SNAI1 signal (P<0.05, Fig. 5B). Furthermore, Spearman’s correlation analysis indicated that miR-153 was inversely correlated with SNAI1 expression in PDAC tissues (r=−0.563, P<0.001).

## Discussion

In recent years, it has been reported that microRNAs (miRNAs) regulate carcinogenesis-related gene expression, indicating insight in the initiation and progression of PDAC (25). As more studies show the relationship between miRNAs and PDAC, the potential of miRNAs as novel biomarkers in PDAC is on the increase. Recently, miR-153 was identified as a robust biomarker of oral cancer with a high positive predictive value (12). In the present study, a reduced expression of miR-153 was observed in PDAC cell lines as compared with a normal human pancreatic duct epithelial cell line. We then detected the expression status of miR-153 in samples of surgically resected PDAC tissues and normal pancreas tissues. Our data indicated that the level of miR-153 expression in PDAC tissues was significantly lower than that in normal pancreas tissues. We also investigated the clini-copathological significance of miR-153 expression in PDAC. Statistical analysis indicated that miR-153 was expressed at significantly lower levels in PDAC patients with lymph node metastasis, poor tumor differentiation, tumor recurrence and advanced TNM tumor stage. These results suggest that the downregulation of miR-153 plays critical roles in PDAC progression and development. Accurate prediction of the prognosis for PDAC patients is of great importance, and molecular biomarkers that may serve as prognostic markers are useful in determining an individualized treatment plan for a PDAC patient (26). Our data demonstrate that the low expression of miR-153 was correlated with a significant shorter 3-year OS and RFS for PDAC patients. The univariate and multivariate Cox regression analysis indicated that miR-153 expression was an independent prognostic factor for predicting OS of PDAC patients. Altogether, these results suggest that miR-153 expression is critical for determination of prognosis in PDAC patients.

miR-153 has recently been considered a crucial factor in tumor metastasis (12,15,20). However, the role of miR-153 in PDAC remains to be determined. In the present study, we identified a new role of miR-153 in PDAC. Additionally, we found that the upregulation of miR-153 inhibited cell migration and invasion in MIAPaCa-2 cells. By contrast, the downregulation of miR-153 increased the number of migrated and invaded AsPC-1 cells. These data suggest that miR-153 inhibits PDAC cell migration and invasion. miRNAs exert function by inversely regulating their downstream target genes. SNAI1, which has been considered as a critical pro-metastatic factor in PDAC by inducing EMT (27), is involved in miR-153-mediated EMT in human epithelial cancers (12). Thus, we investigated the regulatory effect of miR-153 on SNAI1 in PDAC cells. The results suggest that, miR-153 inversely regulated SNAI1 abundance in PDAC cells. SNAI1 was also validated as a direct functional target of miR-153 in PDAC. Furthermore, the expression of SNAI1 in PDAC tissues was obviously higher as compared with that in normal pancreas tissues, which was consistent with previous studies (28). A significant inverse correlation between miR-153 and SNAI1 expression was also observed in PDAC tissues. Consequently, we suggest that miR-153 inhibits cell migration and invasion by targeting SNAI1 in PDAC.

In conclusion, we found that miR-153 is downregulated in PDAC and its low expression is associated with poor prognostic features. Moreover, miR-153 expression is an independent prognostic marker for predicting 3-year survival of PDAC patients. *In vitro* studies demonstrate that miR-153 inhibits PDAC cell migration and invasion. Mechanistically, we suggest that miR-153 inhibits PDAC cell migration and invasion by suppressing SNAI1. Taken together, we considered that miR-153 potentially acts as a clinical biomarker, and may also be a therapeutic target in PDAC.

## Figures and Tables

**Figure 1:** Expression of miR-153 in pancreatic ductal adenocarcinoma (PDAC) cases and cells. (A) Comparing differences in the expression levels of miR-153 between PDAC cell lines with different metastatic potentials and the normal human pancreatic duct epithelial cell line HPDE6-C7. n, three independent experiments, ^*^P<0.05. (B) The expression of miR-153 in PDAC tissues was significantly lower than that in normal pancreas tissues. ^*^P<0.05.

**Figure 2:** The overall survival (OS) and recurrence-free survival (RFS) rates were estimated by the Kaplan-Meier method. According to the level of miR-153 expression, Kaplan-Meier 3-year OS and RFS curves of PDAC patients showed that a low expression of miR-153 was significantly correlated with poor prognosis. The median expression value obtained for miR-153 of the 80 PDAC samples detected by RT-qPCR was selected as the cut-off value. PDAC, pancreatic ductal adenocarcinoma.

**Figure 3:** miR-153 reduces the number of migrated and invaded PDAC cells. (A) MIAPaCa-2 cells that were transfected with miR-control (control) and miR-153, respectively, were subjected to RT-qPCR for miR-153 expression. n, three independent experiments, ^*^P<0.05. (B) Cell migration as measured by Boyden chamber assays was inhibited by the upregulation of miR-153 in MIAPaCa-2 cells as compared with the control cells. miR-153-upregulated MIAPaCa-2 cells conferred a fewer number of invaded cells as compared with control cells. n, three independent experiments, ^*^P<0.05. (C) AsPC-1 cells that were transfected with negative control (NC) and miR-153 inhibitor (anti-miR-153), respectively, were subjected to RT-qPCR for miR-153 expression. n, three independent experiments, ^*^P<0.05. (D) Downregulation of miR-153 promoted AsPC-1 cell migration and invasion *in vitro*. n, three independent experiments, ^*^P<0.05. PDAC, pancreatic ductal adenocarcinoma.

**Figure 4:** SNAI1 is identified as a functional target of miR-153 in PDAC. (A) RT-qPCR and (B) western blot analysis of SNAI1 expression in MIAPaCa-2 cells with miR-153 or control vector transfection. n, three independent experiments, ^*^P<0.05. (C) miR-153 and its putative binding sequence in the 3′-UTR of SNAI1. The mutant miR-153 binding site was generated in the complementary site for the seed region of miR-153 (wt, wild-type; mt, mutant type). (D) miR-153 significantly suppressed the luciferase activity that carried wt but not mt 3′-UTR of SNAI1. Anti-miR-153 led to a marked increase in luciferase activity of wt 3′-UTR of SNAI1. n, three repeats with similar results, ^*^P<0.05. PDAC, pancreatic ductal adenocarcinoma; 3′-UTR, 3′-untranslated region.

**Figure 5:** An inverse correlation between miR-153 and SNAI1 expression is observed in PDAC. (A) A comparison of differences in the expression levels of SNAI1 protein between PDAC tissues and normal pancreas tissues was performed. ^*^P<0.05. (B) A significant inverse correlation between miR-153 and SNAI1 expression was observed in PDAC tissues. Representative immunostaining showed a weak expression of SNAI1 in miR-153 high-expressing PDAC tissue and a strong expression of SNAI1 in miR-153 low-expressing tumor. ^*^P<0.05. Scale bar, 50 *µ*m. PDAC, pancreatic ductal adenocarcinoma.

**Table I:** Correlation between the clinicopathological characteristics and miR-153 expression in PDAC.

Characteristics	Total no. of patients, n=80	miR-153 expression		P-value
		Low	High	
Age (years)				0.348
≤60	28	16	12	
>60	52	24	28	
Gender				0.813
Male	27	14	13	
Female	53	26	27	
Tumor margin				0.179
Negative	38	16	22	
Positive	42	24	18	
Lymph node metastasis				0.014^a^
Absent	43	16	27	
Present	37	24	13	
Tumor size (cm)				0.446
≤2	21	9	12	
>2	59	31	28	
Neural invasion				0.496
Negative	33	15	18	
Positive	47	25	22	
Tumor recurrence				0.004^a^
None	39	13	26	
Local and regional metastasis	41	27	14	
Tumor differentiation				0.024^a^
Wel/moderate	34	12	22	
Poor	46	28	18	
Tumor stage				0.001^a^
I+II	39	12	27	
III+IV	41	28	13	

a Statistically significant. PDAC, pancreatic ductal adenocarcinoma.

**Table II:** Univariate and multivariate survival analysis (Cox regression model) for overall survival of the PDAC patients (n=80).

Variables	HR (95% CI)	P-value
Univariate		
Gender (male vs. female)	0.749 (0.339–1.652)	0.474
Age (years) (>60 vs. ≤60)	1.846 (0.694–4.908)	0.219
Tumor size (cm) (>2 vs. ≤2)	1.092 (0.500–2.386)	0.824
Tumor differentiation (poor vs. well + moderate)	3.233 (1.654–4.265)	0.013^a^
Tumor stage (III+IV vs. I+II)	2.989 (1.678–3.476)	0.015^a^
Tumor margin (positive vs. negative)	0.411 (0.160–1.056)	0.065
Lymph node metastasis (present vs. absent)	1.603 (1.123–2.551)	0.034^a^
Neural invasion (positive vs. negative)	2.113 (0.888–5.030)	0.091
Tumor recurrence (local and regional metastasis vs. none)	1.875 (1.123–3.522)	0.026^a^
miR-153 expression (low vs. high)	2.652 (1.459–3.188)	0.008^a^
Multivariate		
Tumor size (cm) (>2 vs. ≤2)	1.670 (0.787–3.545)	0.182
Tumor differentiation (poor vs. well + moderate)	1.031 (0.492–2.162)	0.936
Tumor stage (III+IV vs. I+II)	2.034 (1.398–2.573)	0.005^a^
Tumor margin (positive vs. negative)	1.971 (0.827–4.696)	0.126
Lymph node metastasis (present vs. absent)	2.119 (1.505–2.499)	0.017^a^
Neural invasion (positive vs. negative)	1.892 (0.940–3.808)	0.074
Tumor recurrence (local and regional metastasis vs. none)	3.225 (2.408–4.234)	0.007^a^
miR-153 expression (low vs. high)	4.123 (2.456–5.033)	0.038^a^

HR, hazard ratio; CI, confidence interval.

a Statistically significant. PDAC, pancreatic ductal adenocarcinoma.
